The article "Scutellarin Loaded on Ultradeformable Nanoliposome Scutellarin EDTMP (S-UNL-E) Promotes Osteogenesis in Osteoporotic Rats" was retracted in 2023. Reasons: signs of a paper mill; suspected computer-generated content; unreliable results or conclusions; lack of ethics approval or compliance.

# Scutellarin Loaded on Ultradeformable Nanoliposome Scutellarin EDTMP (S-UNL-E) Promotes Osteogenesis in Osteoporotic Rats

**DOI:** 10.1155/2022/1395299

**Published:** 2022-08-16

**Authors:** Minhua Teng, Xiao Yuan, Dashan Wang, Hui Gao, Kaiyue Zhang, Wenxue Wang, Baodong Zhao

**Affiliations:** ^1^Department of Oral Implantology, The Affiliated Hospital of Qingdao University, Qingdao 266000, China; ^2^School of Stomatology, Qingdao University, Qingdao 266003, China; ^3^Department of Orthodontics, The Affiliated Hospital of Qingdao University, Qingdao 266000, China

## Abstract

Scutellarin is known as a safe, effective, and low-cost traditional Chinese medicine and has a variety of biological activities. Studies reported that the scutellarin loaded on ultradeformable nanoliposome scutellarin EDTMP (S-UNL-E) could promote osteoblast differentiation and bone formation in vitro. However, its effect on promoting osteogenesis in vivo is still unclear. In this study, pharmacology network and transcriptome sequencing were used to screen the potential targets and pathways of scutellarin in treating osteoporosis. The female Sprague-Dawley (SD) rats were operated on with bilateral oophorectomy and femoral defect to establish an osteoporosis model and then treated separately with bone dust, single scutellarin, 40 mg/kg ultradeformable nanoliposome scutellarin (S-UNL), and the optimal concentration of 40 mg/kg S-UNL-E for a total of 56 d to detect the parameters of trabecular bones. And qRT-PCR and western blot were performed to determine the expression of prostaglandin-endoperoxide synthase 2 (PTGS2), alkaline phosphatase (ALP), transcription factor 4 (TCF4), and *β*-catenin. Results of microscopic computed tomography (Micro-CT) of trabecular bones showed that single scutellarin, S-UNL, and S-UNL-E all promoted the bone formation of osteoporotic rats, in which S-UNL-E manifested the most remarkable therapeutic effect. And it is found that 40 mg/kg of S-UNL-E increased the expression of PTGS2, ALP, TCF4, and *β*-catenin, which indicated that S-UNL-E stimulated the secretion of ALP in bone defect areas to promote bone healing, and increased PTGS2 expression thereby enhancing the transcription and translation of key gene *β*-catenin and TCF4 in the Wnt/*β*-catenin signaling pathway to treat osteoporotic rats.

## 1. Introduction

Scutellarin seems as a safe, effective, and low-cost traditional Chinese medicine, which has a variety of biological activities, such as dilating microvessels, reducing blood viscosity, increasing cerebral blood flow, improving microcirculation, improving lipid metabolism, anti-inflammation, antiapoptosis, antioxidation, and antiallergy [1–3]. Recent studies have shown that scutellarin could treat osteoporosis by upregulating BMP2 transcriptional activity and mRNA expression level to induce osteogenic differentiation via activating the BMP pathway and by inhibiting osteoclast differentiation by negatively regulating RANKL-mediated MAPKs and NF-*κ*B signaling pathway [4]. Another study proved that scutellarin could promote the proliferation and differentiation of human osteoblasts in a short time. With the concentration increase of scutellarin, osteoblast proliferation increased. And scutellarin increased the activity of osteoblasts by promoting alkaline phosphatase (ALP) secretion with dose dependence [5]. In addition, scutellarin increased expression of CXCR4 in osteoporotic rats, which is involved in bone remodeling [6].

The article "Scutellarin Loaded on Ultradeformable Nanoliposome Scutellarin EDTMP (S-UNL-E) Promotes Osteogenesis in Osteoporotic Rats" was retracted in 2023. Reasons: signs of a paper mill; suspected computer-generated content; unreliable results or conclusions; lack of ethics approval or compliance.

With the development of the study on the osteogenic properties of scutellarin, it is expected to be used in the treatment of bone defects in edentulous areas. But it is difficult to deliver drugs to the lesion according to the traditional way of administration due to the biological characteristics of high hardness, poor permeability, and low blood flow of bone tissue. And the shortcomings of low curative effect and severe adverse reactions are ubiquitous in systemic administration in the treatment of bone-related diseases. In recent years, a drug delivery system with a particle size of 1-1000 nm has been developed by using nanotechnology to produce carrier materials and drugs, which can form new controlled drug release agents, reduce the possible toxic and side effects of drugs, achieve drug sustained-release and targeting, and avoid premature diffusion and clearance of drugs [7, 8]. The concept of “bone targeting” means that compound molecules tend to be deposited in bone and incorporated with hydroxyapatite, which can bind to bone calcium. The representative compound ethylenediamine tetramethylphosphonic acid (EDTMP) has been widely studied and applied as a bone target carrier of radionuclides. In the previous study, ultradeformable nanoliposome scutellarin EDTMP (S-UNL-E) was successfully prepared and its osteogenesis function with different concentrations in vitro has been demonstrated. That is, S-UNL-E increased the expression of ALP and the content of osteocalcin, which promoted the ability of osteoblasts to form mineralized nodules [9].

The purpose of this study was to determine the therapeutic effect of S-UNL-E in treating osteoporotic rats and to figure out its mechanism. This study used pharmacology network and transcriptome sequencing to screen the potential targets and pathways of scutellarin in treating osteoporosis. Our results demonstrated the effect of S-NUL-E in treating poor bone mass and its mechanism of action, which could provide a new solution for clinical therapy of bone defects.

The article "Scutellarin Loaded on Ultradeformable Nanoliposome Scutellarin EDTMP (S-UNL-E) Promotes Osteogenesis in Osteoporotic Rats" was retracted in 2023. Reasons: signs of a paper mill; suspected computer-generated content; unreliable results or conclusions; lack of ethics approval or compliance.

## 2. Methods

### 2.1. Network Pharmacology Analysis

PubChem database (https://pubchem.ncbi.nlm.nih.gov) and SwissTarget database (http://old.swisstargetprediction.ch/) were used to predict targets of scutellarin. The targets of osteoporosis were obtained from GeneCards (http://www.genecards.org). Then, Sangerbox (http://sangerbox.com) and STRING (https://www.string-db.org/) were adopted for Venn diagram and protein-protein interaction (PPI) network graphing. Next, Database of Annotation, Visualization and Integrated Discovery (DAVID) (https://david.ncifcrf.gov) was used for KEGG enrichment analysis of the overlapped genes.

### 2.2. Preparation of S-UNL-E

The preparation methods of ultradeformable nanoliposome scutellarin (S-UNL) and S-UNL-E were conducted as described in a previous study [9].

### 2.3. Cell Culture and Grouping

The isolation, culture, purification, and passage of osteoblasts were conducted as in our previous study [9]. Osteoblasts were divided into 5 groups. The control group was treated with complete DMEM; the scutellarin group was treated with single scutellarin; groups of S-UNL-E-7, S-UNL-E-8, and S-UNL-E-9 were treated with S-UNL-E based on the concentrations 2.5 × 10^7^, 2.5 × 10^8^, and 2.5 × 10^9^, separately. Twelve hours after treatment, cells were then collected for subsequent qRT-PCR and western blot tests.

### 2.4. Animal Grouping and Fluorescence Labeling

The animal study was approved by the Committee on the Ethics of Animal Experiments of the Affiliated Hospital of Qingdao University. Twenty-five 12-week-old female SD rats were purchased from Ensiweier Co., Ltd (Chongqing, China). After adaptive feeding for 10 d, rats were randomly divided into a sham group, model group, scutellarin group, S-UNL group, and S-UNL-E group evenly. Except for the sham group, bilateral ovariectomy was performed in rats. Then, those animals were fed for 4 weeks, and the ovariectomized rats were subsequently subjected to bulk bone defects (6 × 1 × 1 mm) in the distal femur to establish an osteoporosis model. The control group and model group received artificial bone dust and intraperitoneal injection of 0.9% normal saline; the scutellarin group received artificial bone dust and scutellarin 40 mg/kg per day; the S-UNL group received artificial bone dust and S-UNL 40 mg/kg per day; the S-UNL-E group received artificial bone dust and S-UNL-E 40 mg/kg per day. The optimum concentration of scutellarin used in the present experiment was with reference to the previous study [6]. Then, rats were treated for a total of 8 weeks.

The article "Scutellarin Loaded on Ultradeformable Nanoliposome Scutellarin EDTMP (S-UNL-E) Promotes Osteogenesis in Osteoporotic Rats" was retracted in 2023. Reasons: signs of a paper mill; suspected computer-generated content; unreliable results or conclusions; lack of ethics approval or compliance.

### 2.5. Microscopic Computed Tomography (Micro-CT) and Data Analysis

Eight weeks after the operation, the distal femur bones of the rats were removed under aseptic conditions, and samples were prepared along the edge of the defect area by 2 mm. To figure out the new bone formation at the bone defects, all samples were scanned and analyzed by Micro-CT. The sample was put into a 2 mL cryopreservation tube and injected 4% paraformaldehyde fixative solution to prevent them from drying. The tubes were then placed vertically into the sample cylinder, and the gap between the tubes was filled with soft sponges to keep the tubes stable during scanning. Next, the sample cylinder was put into the Micro-CT sample rack (SkyScan 1276, Bruker, USA). The scanning range of each sample was determined to be within 3 mm of the upper and lower margins of the femoral defect. In order to obtain the maximum signal to noise ratio (SNR), the high-resolution scanning mode was selected. The scanning parameters were set as follows: 70 kV of bulb voltage, 114 mA of scanning current, and 70 ms of integration time. During 3D reconstruction and quantitative analysis, Gaussian filter parameters were set as *σ* = 1.2, support = 1, and bone tissue threshold = 205 − 700. The parameters related to the microscopic quantitative analysis of trabecular bones were as follows: relative bone volume (bone volume/total volume, BV/TV), trabecular thickness (Tb.Th, mm), trabecular number (Tb.N, mm^−1^), connectivity density (Conn.D, mm^−3^), and trabecular separation (Tb.Sp, mm).

### 2.6. Transcriptome Sequencing

The transcriptome sequencing was supported by Biomedicine Biotech Co., Ltd, Chongqing, China. Osteoblasts of rats in the control group and S-UNL-E group were used to extract RNA separately for transcriptome sequencing. The library was prepared by TruSeq® Stranded Total RNA Library Prep kit (#20020596, Illumina, USA). The purity, concentration, and integrity of RNA were detected by a nanophotometer (N60, Implen, Germany), Qubit® 3.0 Fluorometer (Q33216, Life Technologies, USA), and RNA Agilent 6000 Nano Kit (#5067-1511, Agilent, USA), respectively. Illumina HiSeq2500 system (USA) was used for sequencing. FastQC software (version 0.11.9, UK) was used to control the quality of RNA sequences, and the known Illumina TruSeq joint sequences, low mass sequences, and ribosomal RNA sequences were removed. Hisat2 (version 2.2.1, USA) was then used to map the reserved sequence to the rat reference genome, and StringTie (version 2.2.0, USA) was used to screen every gene count in the reserved sequence, and gene count was normalized with TMM of EdgeR (version 3.14, USA) [10]. FPKM value was calculated with Perl scripts [11]. Differentially expressed genes (DEGs) were analyzed by EdgeR [12]. And *p* value < 0.05 and |log2FoldChange| > 1 were used as the criterion of significant difference [13]. Venny was used to screen for highly expressed DEGs. ClusterProfiler (version 4.0.3, USA) was applied for GO and KEGG enrichment analysis.

The article "Scutellarin Loaded on Ultradeformable Nanoliposome Scutellarin EDTMP (S-UNL-E) Promotes Osteogenesis in Osteoporotic Rats" was retracted in 2023. Reasons: signs of a paper mill; suspected computer-generated content; unreliable results or conclusions; lack of ethics approval or compliance.

### 2.7. qRT-PCR

Total cellular RNA of osteoblasts from rats was extracted by Trizol (#15596026, Invitrogen, USA) following the instruction. The reverse transcription was carried out with Goldenstar RT6 cDNA Synthesis Kit (TSK302M, Tsingke, Beijing, China). An RNase-free EP tube was prepared, and gDNA remover, 10× gDNA remover Buffer, dNTP Mix, Oligo dT, Randomer, DTT, and RT6 were added with 1 *μ*L, respectively. Then, 2 *μ*L of total RNA, 4 *μ*L of 5× Goldenstar™ Buffer, and 7 *μ*L of RNase-Free ddH_2_O were added. The reaction was performed on the platform of a thermal cycler instrument (T100, Bio-Rad, USA). Reaction conditions defaulted at 25°C for 10 min, 55°C for 50 min, and 85°C for 5 min. According to the instructions of 2× T5 Fast qPCR Mix (TSE002, Tsingke, Beijing, China), qPCR reaction system was settled as follows: 0.4 *μ*L of 50× ROX Reference Dye II, 0.5 *μ*L of template, 0.8 *μ*L of forward primer, 0.8 *μ*L of reverse primer, 10 *μ*L of 2× T5 Fast qPCR Mix, and 7.5 *μ*L of RNase Free dH_2_O. Next, the reaction conditions were adjusted at 95°C for 30 s, followed at 95°C for 5 s, and 55°C for 30 s, 40 cycles in total, subsequently from 72°C for 30 s, and performed with CFX7500 real-time fluorescence quantitative instrument (Bio-Rad, USA). The primer sequences were shown as follows: PTGS2 (COX2)-F, AGGAGCATCCTGAGTGGGAT; PTGS2 (COX2)-R, TTCAGAGGCAATGCGGTTCT; *β*-catenin-F, ACTCTGAGAAACTTGTCCGATGC; *β*-catenin-R, AGATGGCAGGCTCGGTAATG; TCF4-F, ATGGAGCAATGGGCAGTC; TCF4-R, GGGTGGGTTCAAGTCAGG; ALP-F, CAGTGGTATTGTAGGTGCTGTG; ALP-R, TTTCTGCTTGAGGTTGAGGTTAC; GAPDH-F, GCAAGTTCAACGGCACAG; GAPDH-R, GCCAGTAGACTCCACGACATA.

### 2.8. Western Blot

Cellular protein of osteoblasts from rats was extracted with RIPA lysis buffer (#P0013B, Beyotime, China), and BCA kit (#P0012S, Beyotime, China) was adopted to determine the protein concentration. Subsequently, the SDS-PAGE gels were prepared according to the SDS-PAGE kit (#PG112, Epizyme, China). The electrophoresis condition was set at 80 V for 1 h and then was adjusted to 120 V for 40 min. The membrane transfer condition was settled at 250 mA for 2 h. Then, 5% skimmed milk was used for blocking at 25°C for 1 h. Primary antibodies PTGS2 (#A1253, ABclonal, China), *β*-catenin (#A19657, ABclonal, China), TCF4 (#A1141, ABclonal, China), ALP (#A19286, ABclonal, China), and GAPDH (#A19056, ABclonal, China) (dilutions of 1 : 1000, 1 : 500, 1 : 500, 1 : 500, and 1 : 100, respectively) were added for incubation overnight at 4°C. The membranes were washed 3 times with TBST, 10 min each time. Next, secondary antibody (#AS014, ABclonal, China) was added to the membranes and incubated at room temperature for 1 h. Then, the membranes were rinsed with TBST 3 times, 10 min each time, and exposed using ECL exposure liquid. The gray values of the target bands were analyzed and calculated by ImageJ (version 1.8.0, USA).

The article "Scutellarin Loaded on Ultradeformable Nanoliposome Scutellarin EDTMP (S-UNL-E) Promotes Osteogenesis in Osteoporotic Rats" was retracted in 2023. Reasons: signs of a paper mill; suspected computer-generated content; unreliable results or conclusions; lack of ethics approval or compliance.

### 2.9. Statistical Analysis

GraphPad Prism (version 9.0, USA) was used for statistical analysis and graphing. The results were expressed as mean ± SD. Mean analysis of multiple groups was subjected to one-way ANOVA methods. The values of *p* < 0.05 indicated that the difference was statistically significant.

## 3. Results

### 3.1. Results of Network Pharmacology Analysis

The potential target genes were predicted by PubMed and SwissTarget databases; there were a total of 100 targets. Then, the targets of scutellarin were intersected with 4273 osteoporosis targets in GeneCards database, and there were 58 overlapped genes in total (Figure 1(a)). According to PPI network, the more interactions between two proteins, the more connections. And considering the purpose of the present study, PTGS2 was selected as the candidate gene for the following experiments (Figure 1(b)). To clarify the functions and signaling pathways of the overlapped genes, DAVID database was used to perform KEGG enrichment analysis. A total of 23 signaling pathways were obtained, and the top 6 pathways were as follows: pathways in cancer, TNF signaling pathway, proteoglycans in cancer pathway, MAPK signaling pathway, HTLV-I infection pathway, and microRNAs in cancer pathway (Table 1).

### 3.2. DEG Analysis in Rats after S-UNL-E Administration

To understand the mechanisms of S-UNL-E on osteoporosis in-depth, RNA sequencing analysis was performed to obtain the mRNA expression levels of the samples. In general, the number of DEGs only accounts for a small fraction of the overall genes, and a small number of DEGs do not have much effect on the expression distribution of the samples. So, all samples should have similar expression distribution. Based on the gene expression of all samples, a heat map of DEGs was obtained (Figure 2(a)). A total of 2911 DEGs were screened by bioinformatics analysis. There were 1949 down-DEGs in the control group and 962 reversed down-DEGs in the S-UNL-E group (Figure 2(b)). Then, GO enrichment analysis and KEGG enrichment analysis were performed by ClusterProfiler. Down-DEGs were mainly enriched in the items of extracellular matrix, muscle structure development, tissue morphogenesis, skeletal system development, and response to wounding with GO analysis, and KEGG pathways were mainly enriched in human papillomavirus infection, PI3K-Akt signaling pathway, and focal adhesion (Figures 3(a) and 3(c)). The top 5 results of GO analysis of reversed down-DEGs were cellular cation homeostasis, cellular ion homeostasis, metal ion homeostasis, response to bacterium, and cation homeostasis (Figure 3(b)); the top 3 KEGG pathways were PI3K-Akt signaling pathway, cytokine-cytokine receptor interaction, and chemokine signaling pathway (Figure 3(d)).

The article "Scutellarin Loaded on Ultradeformable Nanoliposome Scutellarin EDTMP (S-UNL-E) Promotes Osteogenesis in Osteoporotic Rats" was retracted in 2023. Reasons: signs of a paper mill; suspected computer-generated content; unreliable results or conclusions; lack of ethics approval or compliance.

### 3.3. Effect of S-UNL-E on the Expression of Genes Related to Osteoblast Differentiation

In this experiment, cells were divided into three groups and treated with 2 × 10^7^, 2 × 10^8^, and 2 × 10^9^ S-UNL-E, respectively. Results in vitro showed that both scutellarin and S-UNL-E significantly increased the mRNA expressions (Figures 4(a)–4(d)) and protein expressions (Figures 4(e)–4(i)) of PTGS2, *β*-catenin, TCF4, and ALP in osteoblasts compared to the control group, and the difference in the S-UNL-E-8 group turned the most remarkable versus other groups.

### 3.4. Effect of S-UNL-E on Bone Formation in Osteoporotic Rats

After 56 d of administration, the trabecular bones of rats were collected for parameter analysis. BV/TV, Tb.Th, Tb.N, and Conn.D were markedly decreased, and Tb. SP was significantly increased in the model group compared to the control group (Figures 5(a)–5(e)). However, in scutellarin-, S-UNL- and S-UNL-E-treated groups, the parameters were all contrary to the model group, in which the S-UNL-E group manifested the most remarkable therapeutic effect.

### 3.5. Effect of S-UNL-E on Osteogenetic-Related Gene Expression in Rats

Results in vivo manifested the same tendency of the expression of PTGS2, *β*-catenin, TCF4, and ALP. The indices in model groups decreased significantly versus the sham operation group (Figures 6(a)–6(d)). But when rats were treated for 56 d with the optimum concentration of S-UNL and S-UNL-E, the protein expressions were all markedly higher than the model group, even significantly higher than the sham operation group (Figures 6(e)–6(i)). And the S-UNL-E group still manifested the most remarkable curative effect among all scutellarin treatment groups.

## 4. Discussion

### 4.1. S-UNL-E Promoted Bone Healing in Ovariectomized Rats

The development of scutellarin, a traditional Chinese medicine, as a treatment for a series of diseases such as cerebral and myocardial ischemia, diabetes, neurodegeneration, and cancer has become a promising treatment direction. And advanced studies proved its functions in bone formation and osteogenesis, providing a new potential therapy method in the field of oral implants. But the defects of traditional administration methods bring challenges in delivering drugs to the lesions, and new drug delivery systems need to be developed. In our previous study, scutellarin loaded on ultradeformable nanoliposome scutellarin EDTMP was prepared with nanotechnology, which has the characteristics of active and passive dual targeting. And the results demonstrated that S-UNL-E promoted osteogenic differentiation and bone formation in vitro. To investigate the therapeutic effect in animal models in depth, the potential overlapped target genes between scutellarin and osteoporosis were predicted through pharmacology network and thus providing the research basis of this study.

The article "Scutellarin Loaded on Ultradeformable Nanoliposome Scutellarin EDTMP (S-UNL-E) Promotes Osteogenesis in Osteoporotic Rats" was retracted in 2023. Reasons: signs of a paper mill; suspected computer-generated content; unreliable results or conclusions; lack of ethics approval or compliance.

Osteoporosis is associated with ovarian dysfunction, and the decrease in estrogen level is considered an important factor resulting in osteoporosis [14, 15]. Bone formation and differentiation are affected by the expression of estrogen receptors in bone tissue. When the estrogen level decreases, the risk of bone fracture increases, as well as the bone density decreases and bone microstructure deteriorates [16]. Therefore, bilateral ovariectomy and femoral defect were operated on to establish osteoporosis model rats. And the rats in different groups were treated with artificial bone dust, 40 mg/kg S-UNL, 40 mg/kg S-UNL-E, and single scutellarin for 56 d and then performed the subsequent experiments. Result of Micro-CT showed that the relative bone volume, trabecular thickness, trabecular number, and bone connectivity density were all increased, and trabecular separation was decreased in the three groups containing scutellarin compared with the model group. Moreover, the treatment effect of S-UNL-E was better than that of the S-UNL group or single scutellarin group, which indicated that scutellarin could promote the differentiation of osteoblasts in vivo. Furthermore, when scutellarin is delivered by EDTMP, it could target the lesion and achieve a superior therapeutic effect.

### 4.2. S-UNL-E Increased PTSG2, *β*-Catenin, TCF4, and ALP Expressions to Enhance Osteogenesis

With the purpose of examining the mechanism of S-UNL-E in treating osteoporosis, PTGS2, *β*-catenin, TCF4, and ALP were selected for deeply studying based on pharmacology network and transcriptome sequencing technology. PTGS2, also known as cyclooxygenase 2 (COX-2), is considered a biomarker and osteogenic enhancer of glucocorticoid-induced osteonecrosis of the femoral head. Its expression in inflammation can promote osteoblast differentiation of mesenchymal stem cells [17]. Prior studies identified that PTGS2 was involved simultaneously in osteogenesis [18] and highly expressed in human osteoarthritis chondrocytes [19]. PTGS2 also plays a key role in the differentiation of mesenchymal stem cells into osteoblast cell lines and osteoclast maturation [20]. The Wnt/*β*-catenin pathway regulates osteogenic differentiation, bone formation, and bone metabolic disorders in bone marrow mesenchymal stem cells [21–24]. And transcription factor 4 (TCF-4), one of the main members of the TCF/LEF family, is a basic helix-loop helix transcription factor with dual regulatory effects and plays an important role in Wnt/*β*-catenin signaling pathway. TCF4 can binds to *β*-catenin in the nucleus to jointly regulate and activate transcription of its downstream target genes [25]. ALP is a marker enzyme on biofilm, which exists in organs such as bone, liver, kidney, and small intestine. ALP secreted by osteoblasts can be used as a specific biomarker to detect osteoblast differentiation. When the process of bone formation is hyperactive, osteoblasts proliferate significantly and ALP is secreted in large quantities [26]. In this study, it is found that S-UNL-E increased the expression of ALP to stimulate the secretion of ALP in bone defect area to promote the bone formation. Furthermore, S-UNL-E promoted the expression of PTGS2, *β*-catenin, and TCF4 both in vitro and in vivo, which indicated that S-UNL-E increased the PTGS2 expression thereby promoting the transcription and translation of key gene *β*-catenin and TCF4 in the Wnt/*β*-catenin signaling pathway to treat osteoporosis. And above all the concentrations of S-UNL-E, 2 × 10^8^ (40 mg/kg) achieved the best effect on osteoblast differentiation and bone healing.

The article "Scutellarin Loaded on Ultradeformable Nanoliposome Scutellarin EDTMP (S-UNL-E) Promotes Osteogenesis in Osteoporotic Rats" was retracted in 2023. Reasons: signs of a paper mill; suspected computer-generated content; unreliable results or conclusions; lack of ethics approval or compliance.

## 5. Conclusion

S-UNL-E increased the expression of PTGS2 to promote the transcription and translation of key genes *β*-catenin and TCF4 in the Wnt/*β*-catenin signaling pathway, and S-UNL-E promoted the expression of ALP gene, leading to excessive secretion of ALP by osteoblasts, thereby together promoting osteoblast

## Figures and Tables

**Figure 1:** Target genes of scutellarin for the treatment of osteoporosis based on network pharmacology analysis. (a) Venn diagram of overlapped genes. (b) PPI network of overlapped genes.

**Figure 2:** Bioinformatics analysis of DEGs. (a) Heat map. The horizontal coordinates are the samples, and the vertical coordinates are the normalized values of the differential gene FPKM. The redder the color, the higher the expression, and the greener the color, the lower the expression. (b) Volcano map. The horizontal coordinates are the log2FoldChange values, the vertical coordinates are −log10*p*adj values, and the blue dashed line indicates the threshold line for the DEG screening criteria. SE: S-UNL-E group; NC: sham group.

The article "Scutellarin Loaded on Ultradeformable Nanoliposome Scutellarin EDTMP (S-UNL-E) Promotes Osteogenesis in Osteoporotic Rats" was retracted in 2023. Reasons: signs of a paper mill; suspected computer-generated content; unreliable results or conclusions; lack of ethics approval or compliance.

**Figure 3:** GO and KEGG enrichment analysis of DEGs. (a) GO enrichment analysis of down-DEGs. (b) GO enrichment analysis of reversed down-DEGs. (c) KEGG enrichment analysis of down-DEGs. (d) KEGG enrichment analysis of reversed down-DEGs. The horizontal coordinates are the ratio of the number of DEGs to the total number of DEGs that are annotated to GO/KEGG terms, and the vertical coordinates are the GO/KEGG terms.

**Figure 4:** Relative mRNA and protein expressions of PTGS2, *β*-catenin, TCF4, and ALP after osteoblasts were treated with 2 × 10^7^, 2 × 10^8^, and 2 × 10^9^ S-UNL-E. (a–d) The mRNA levels were analyzed by qRT-PCR. (e) The expression levels were analyzed by western blot. (f–i) The western blot results were qualified. ^∗∗∗^*p* < 0.001*vs.* control.

**Figure 5:** SUN-L-E promoted the bone healing in osteoporotic rats. (a) BV/TV (%). (b) Tb.Th (mm). (c) Tb.N (mm^−1^). (d) Conn.D (mm^−3^). (e) Tb.Sp (mm). ^∗∗^*p* < 0.01 and ^∗∗∗^*p* < 0.001*vs.* sham. ^#^*p* < 0.05, ^##^*p* < 0.01, and ^###^*p* < 0.001*vs.* model.

**Figure 6:** Relative mRNA and protein expressions of PTGS2, *β*-catenin, TCF4, and ALP of rats after being treated with 40 mg/kg S-UNL-E. (a–d) The mRNA levels were analyzed by qRT-PCR. (e) The expression levels were analyzed by western blot. (f–i) The western blot results were qualified. ^∗^*p* < 0.05, ^∗∗^*p* < 0.01, and ^∗∗∗^*p* < 0.001*vs.* sham. ^#^*p* < 0.05, ^##^*p* < 0.01, and ^##^*p* < 0.001*vs.* model.

**Table 1:** DAVID analysis of overlapped genes.

Term	Count	%	Genes
Pathways in cancer	5	20.84	FLT3, CASP3, KIT, PTGS2, HRAS
TNF signaling pathway	4	16.67	CASP7, CASP3, PTGS2, TNF
Proteoglycans in cancer	4	16.67	CASP3, HRAS, ESR1, TNF
MAPK signaling pathway	4	16.67	RPS6KA3, CASP3, HRAS, TNF
HTLV-I infection	4	16.67	TERT, HRAS, TNF, IL2
MicroRNAs in cancer	4	16.67	CASP3, CYP1B1, PTGS2, HRAS
Ovarian steroidogenesis	3	12.50	CYP1A1, CYP1B1, PTGS2
Legionellosis	3	12.50	CASP7, CASP3, TNF
Acute myeloid leukemia	3	12.50	FLT3, KIT, HRAS
Apoptosis	3	12.50	CASP7, CASP3, TNF
Central carbon metabolism in cancer	3	12.50	FLT3, KIT, HRAS
Pertussis	3	12.50	CASP7, CASP3, TNF
Chemical carcinogenesis	3	12.50	CYP1A1, CYP1B1, PTGS2
Hematopoietic cell lineage	3	12.50	FLT3, KIT, TNF
Estrogen signaling pathway	3	12.50	OPRM1, HRAS, ESR1
T cell receptor signaling pathway	3	12.50	HRAS, TNF, IL2
Serotonergic synapse	3	12.50	CASP3, PTGS2, HRAS
Sphingolipid signaling pathway	3	12.50	OPRD1, HRAS, TNF
Natural killer cell-mediated cytotoxicity	3	12.50	CASP3, HRAS, TNF
Hepatitis B	3	12.50	CASP3, HRAS, TNF
Nonalcoholic fatty liver disease (NAFLD)	3	12.50	CASP7, CASP3, TNF
Alzheimer's disease	3	12.50	CASP7, CASP3, TNF
Graft-versus-host disease	2	8.33	TNF, IL2

The article "Scutellarin Loaded on Ultradeformable Nanoliposome Scutellarin EDTMP (S-UNL-E) Promotes Osteogenesis in Osteoporotic Rats" was retracted in 2023. Reasons: signs of a paper mill; suspected computer-generated content; unreliable results or conclusions; lack of ethics approval or compliance.

## Data Availability

All data, models, and code generated or used during the study appear in the submitted article.

## Additional Points

*Highlights*. 40 mg/kg S-UNL-E promoted osteoblast differentiation and bone formation in osteoporotic rats. 40 mg/kg S-UNL-E promoted the expression of ALP gene to secrete excessive ALP by osteoblasts. 40 mg/kg S-UNL-E promoted the expression of PTGS2 to activate the Wnt/*β*-catenin signaling pathway.
